# The Role of Music Therapy in the Emotional Regulation and Psychological Stress Relief of Employees in the Workplace

**DOI:** 10.1155/2022/4260904

**Published:** 2022-01-29

**Authors:** Nan Mao

**Affiliations:** Music Department, Xi'an Shiyou University, Xi'an 710065, Shanxi, China

## Abstract

With the increasing global attention to the problem of staff stress, scholars in the fields of sociology, psychology, and medicine are seeking effective solutions. Music therapy has entered the field of vision of scholars with its unique advantages and is used to maintain the mental health of workers in various industries and improve work efficiency. To solve the problem of employees' psychological pressure, ordinary psychotherapy is mainly done through conversation. At present, the psychological pressure generated by employees in the workplace is obviously unable to be treated by ordinary psychological treatment methods. Music therapy can play its role in this situation. This article collects a large amount of data through surveys to obtain the job satisfaction data of medical care, education, and restaurant staff for the corresponding occupations, analyzes the data, and considers the role of music therapy in this type of industry to relieve the psychological pressure of relevant staff. In the end, it is concluded that music therapy can stimulate employees' creative inspiration, eliminate employee fatigue, and eliminate some potential unfavorable factors. It can also enhance the friendship between employees, improve employee work efficiency and employees' sense of corporate identity, and reduce employee pain sense. In general, music therapy can have a positive impact in many areas, especially in corporate applications, which can have a positive impact on employees in many aspects in the workplace.

## 1. Introduction

### 1.1. Workplace Stress

In the Internet age, most industries have achieved programmatic management, but the work pressure in all walks of life is not less than that of physical activity work in the early twentieth century [1]. The results of the ILO's research show that there are 10 companies in every part of the world [2] in which one of the employees suffers from anxiety, depression, physical exhaustion, and stress. Long time work pressure may even lead to depression, which has a huge negative impact on the physical and mental health of employees [3]. In detail, work stress is a kind of complex emotions generated by employees for complex tasks under the influence of a variety of uncertain factors [4]. There are many reasons for stress, including worry about unknown and difficult tasks, long overtime work that leads to mental stress, worry about the effects of sedentary on the body, scientific and technological progress, the fear of new knowledge in the industry, office politics [5], and worries about being replaced by future automation technology or robots [6]. From the above reasons, it can be seen that there are many kinds of work pressures for modern office employees [7]. Under pressure, the work efficiency of employees will be greatly reduced [8]. From a macro point of view, the production efficiency of enterprises will be reduced [9]. It will also reduce the productivity of society. Therefore, it is urgent to find a way to deal with the pressure of employees in the workplace. Music therapy can help relieve pain, help focus, improve athletic performance, improve mood, and make people feel at ease. This article first analyzes the necessity of applying music therapy to psychological adjustment of employees in workplace, then analyzed different effects of music therapy on employees' emotion regulation, and finally summarized the role of music therapy in the psychological stress relief of employees in different workplaces.

### 1.2. Definition of Music Therapy

With the increasing global attention to the problem of staff stress, scholars in the fields of sociology, psychology, and medicine are seeking effective solutions. Music therapy has entered the field of vision of scholars with its unique advantages and is used to maintain the mental health of workers in various industries and improve employee productivity. Regarding the definition of music therapy [10], we must first understand the two basic elements of music therapy: treatment target and treatment goals [11]; countries around the world have different definitions of music therapy, but they are inseparable from the two basic elements of treatment target and treatment goals [12]. Mayer defined music therapy in a recent literature as follows: “Music therapy is the use of various ways of music experience to help the person being treated achieve the goal of mental or physical health.” The target of music therapy is mainly graduate students who are about to graduate, industry workers, people with autism, and other groups with psychological and physical needs for treatment [13].

Music therapy is not a random or simple process of playing music. The treatment cycle is divided into short-term and long-term types [14]. The treatment process contains a variety of theories and methods. After determining the treatment target [15], a detailed treatment plan needs to be formulated. Music psychotherapy, as an auxiliary means in psychological counseling, counseling, and activities, is a choice that meets the public's psychological needs and appreciation habits [16].

## 2. The Necessity of Applying Music Therapy to Psychological Adjustment of Employees in Workplace

Compared with ordinary psychotherapy, music therapy has a more significant effect on our staff. Ordinary psychotherapy is mainly done through conversation [17], and music therapy also adds music entertainment functions on this basis. When ordinary psychotherapy is not applicable to the target, music therapy can be used. At present, the psychological stress caused by employees in the workplace is obviously unable to be treated by ordinary psychological treatment methods. Even if this method is adopted [18], the company's operating costs and operating efficiency will be reduced. At present, even in the world's top industry leading company, I have never seen the establishment of a professional employee psychological counseling department, so music therapy can play its unique role in this situation [19].

Ordinary psychotherapeutic programs are mainly to change employees' wrong views on problems for treatment [20]. This program cannot treat psychological problems caused by emotions, while music therapy can improve the emotional state of individuals. The use of various sedative drugs will not only have unknown side effects of dependence [21] but also increase the financial pressure of employees [22]. Music therapy can play corresponding music according to the needs of employees without side effects and is cost-effective, which is very friendly to employees. The comparison of general psychotherapy and music therapy in detail is shown in Table 1.

Music therapy can have a positive impact on employees' psychology and physiology. In terms of psychology, music brings appeal to employees and different music has different effects on employees' mental states [23]. Rap music can soothe people's hearts and inspire an optimistic and positive attitude of employees, while sad music can stimulate employees' nostalgia and imagination. Beautiful and soft music can stabilize the emotions of employees, and calm and soothing music can soothe restless emotions and ease the tension of employees at work [24]. In terms of physiology, after the adjustment of music therapy, the blood circulation of the human body is accelerated and the body is in a state of relaxation and internal repair. The impact of music therapy on employees' psychological and physical aspects is shown in Figure 1.

## 3. Different Effects of Music Therapy on Employees' Emotion Regulation

Stress is synonymous with the psychological and physiological responses of individuals to various external stimuli. The work pressure is the pressure caused by the reasons that are highly connected to the work. It mainly comes from the external environment, the company, and the individual. Among them, the political, technical, and economic reasons in the external environment can cause pressure in the work, or it may be caused by the inability to complete the corresponding work within the specified time, the content of the work is something that the individual hates, the leader is difficult to get along with, etc., which may cause pressure, and may also be stressed at work due to health condition.

Under short-term external pressure stimulation, the human body will produce reactions such as accelerated breathing, accelerated heart rate, increased blood sugar, increased blood pressure, increased hormone secretion, and nerve excitement. If the duration is not long and the frequency is not high, the human body will not respond harmful effects. However, if you are under high-intensity work pressure for a long time, it will cause many adverse effects. Employees are the blood of the company, and the company will suffer intangible losses. It affects the physical health of employees. Long-term psychological stress can induce many diseases such as coronary heart disease and gastroenteritis. Psychological pressure will cause tension between the employees and superiors of the company, and the employees will not get along well, which will affect the normal operation of the entire team. It may cause low work efficiency and poor quality of completed work content, cause employees to lose interest in work, high absenteeism rate, and ultimately lead to resignation. Direct sources of work stress are shown in Figure 2. In addition to the direct work pressure described in Figure 2, there are also potential pressures in life. These potential pressures may come from drastic changes in the environment, such as the worsening of the epidemic, the illness of relatives and friends, and facing major conference speeches.

### 3.1. Positive Effects of Music Therapy

From this questionnaire, we can see that company employees engaged in mental work and factory employees engaged in manual labor are more inclined to broadcast. The approval rates are as high as 96% and 92%. The way of activities to relieve work pressure is relatively the lowest approval rate, but even the lowest approval rate is 62%, more than half. Therefore, practice shows that the use of music therapy can indeed effectively relieve the work pressure of employees.

#### 3.1.1. Music Therapy Can Inspire Employees to Create Inspiration

When faced with untouched work content, employees will have greater psychological pressure. Music therapy can help employees find solutions to problems and relieve stress. The famous scientist Einstein would pick up his violin when he had no inspiration for writing, and he could always reinvigorate his creative inspiration after a few performances. The same mechanism has been proven in many cases. For challenging work tasks, playing some music that employees like will always allow employees to find creative inspiration.

#### 3.1.2. Music Therapy Can Eliminate Employee Fatigue

Music therapy plays a positive psychological soothing effect on the staff, allowing them to work in a relaxed and comfortable environment, so that the tension formed by the staff in the workplace can be relieved and adjusted. The quality of the work produced by its work will not decline, but on the contrary will be improved to a certain extent.

#### 3.1.3. Music Therapy Eliminates Some Potential Disadvantages

Playing background music in the workplace can eliminate some unfavorable factors in the work, such as employees discussing complicated work processes with customers, discussing special work solutions, and disputes may arise due to disagreements, and the results of the communication may not achieve the desired results of the customers. Unfavorable factors will become the pressure that employees will face in the later stages of the project. However, music therapy can divert the customer's attention and allow customers and employees to communicate with each other in a peaceful state of mind, which makes it easier to reach agreement on cooperation projects.

#### 3.1.4. Music Therapy Can Enhance Friendship among Employees

In the case of the epidemic, employees wear masks and the distrust between each other is strengthened, and even communication is conducted through remote video. Music therapy can solve the psychological pressure problem of employees in this aspect in the later stage of the epidemic. Studies have shown that, under external music therapy, employees are more likely to gain peace of mind, immerse themselves in beautiful and lively music, and thus temporarily forget the psychological pressure caused by work. Studies have shown that it is easier for employees to achieve under stress-free conditions.

#### 3.1.5. Music Therapy Can Improve Employee Productivity

Music therapy allows employees to be in a state of relaxation during work, so that they can maximize their potential, complete the tasks assigned by the leadership with high quality, and improve work efficiency. The most direct reason for their potential is beautiful music. The lively concert promotes the human body to secrete active substances that are beneficial to health and achieve the purpose of regulating the functions of the digestive system, endocrine system, and cardiovascular system. Employees are in a good mental state, and their work efficiency naturally becomes higher.

#### 3.1.6. Music Therapy Can Improve Employees' Sense of Corporate Identity

Excessive psychological pressure on employees in the workplace may reduce employees' sense of identity with the company. Playing beautiful music related to corporate culture in the workplace can relax employees while promoting the company's slogan, thereby realizing employees' psychological stress relief and enhancing employees' sense of corporate identity.

#### 3.1.7. Music Therapy Can Reduce Employee Pain

Researchers used music therapy combined with the comfort-behavior scale and facial expression pain scale to measure the individual's pain after receiving music therapy. Research shows that live music therapy can reduce the individual's pain and suffering.

### 3.2. Negative Effects of Music Therapy

However, music therapy is not all advantageous and it still has certain shortcomings. First, after listening to music at high frequencies uninterrupted, the brain has been paying attention to the music and the nerves are in a long-term state of excitement, which easily makes people feel fatigued, which belongs to the fatigue of excessive excitement. Second, music therapy may distract the subject and affect the logical thinking of the person being treated. There will always be countless inspirations and ideas in the brain. For example, during work, the brain will think of many things and music therapy will seriously affect this. This kind of thinking can also be considered as an influence on creativity. Studies have shown that when doing work that requires a strong logic, playing background music may have a heavy impact on their mind.

## 4. The Role of Music Therapy in the Psychological Stress Relief of Employees in Different Workplaces

Listening to music is a very comfortable thing for most people. However, in the course of music therapy, too loud music may aggravate employees' psychological pressure and too sad music may induce melancholy lurking deep in employees' hearts. Therefore, the workplace should choose some contagious, beautiful sound and slow rhythm music for psychological adjustment, such as Chinese and Western classical music, new century music, and world famous music, which are all good choices.

Different types of music should also be used for treatment for different groups of people. For example, a software development company needs to conduct psychological stress relief music therapy for programmers. The type of music selected cannot be rock or rap music because the programmer's work needs to maintain a sense of logic. The chaotic rhythm can easily disrupt their thoughts about programming. Relatively speaking, light music is more suitable for programmers and the marketing staff of this software development company are suitable for more lively music therapy programs because employees in the marketing department need to communicate with different people in various industries for a long time. Lively music can keep them active and positive. The following will analyze the effect of music therapy on the psychological stress relief of employees in different workplaces. Some scholars collected a large amount of data through interviews to obtain the satisfaction degree of medical care, education, and restaurant staff with the corresponding occupations, as shown in Figure 3.

The study found that employees in the medical, education, and catering industries differ in their satisfaction level with the corresponding occupations. Among them, the highest degree of dissatisfaction is the restaurant and medical industry employees. The dissatisfaction distribution in the surveyed samples has reached 40%, while the education industry workers have a high degree of professional recognition, and their dissatisfaction is less than 25%.

### 4.1. The Effect of Music Therapy on Medical Staff

It can be seen from the chart that when working in a hospital, the mood of doctors is “normal” accounting for 50% of all surveys. 40% of doctors feel “unsatisfied” at work, and only 10% of doctors are satisfied. From another perspective, dissatisfaction and general evaluation are negative views. It can be seen that most doctors have psychological pressure at work. The main reason may be the current tension in the doctor-patient relationship and the doctor's work intensity. It is reported that some surgeons will sometimes work continuously in the operating room for more than ten hours. In this case, the psychological pressure of doctors in the workplace is gradually increasing.

Quiet music helps to eliminate stress. Among them, light music is delicate and expressive, and it has a good effect in the direction of music therapy. If light music is selected for passive piano music therapy for medical staff, music therapists can play suitable light music for medical staff, interspersed with other types of works such as jazz music that can relieve psychological stress. Light music therapy should ultimately achieve the purpose of psychological comfort to medical staff, so as to relieve psychological pressure.

By listening to piano works that soothe the emotions, medical staff can devote themselves to the music scene and finally achieve the purpose of treatment through empathy, that is, to relieve negative emotions and psychological pressure, and maintain a healthy mental state.

### 4.2. The Effect of Music Therapy on Educators

From the chart, we can see that only 20% of teachers are satisfied with their work and 80% of teachers feel fair or dissatisfied. Because of the rapid development and popularization of new media, many teachers' educational behaviors and educational ideas will be actively or passively transmitted to the Internet, resulting in a wider range of dissemination, which will cause greater pressure on teachers.

Studies have shown that after the Nanfang Daily surveyed tens of thousands of teachers in Guangdong Province, it was reported that 94.6% of teachers have psychological pressure, of which 35.6% of teachers have greater psychological pressure. These psychological pressures are gradually affecting teachers' psychology. In relation to physical health, 90% of tens of thousands of teachers are in a subhealth state and 20% of teachers are in a state of illness.

The beautiful and melodious concerts improve the ecological environment of the human body through psychological and physiological channels and create a positive and good living condition. For different psychological problems of different teachers, different types of music should be selected for treatment, such as kindergarten and elementary school teachers. The right student group is in a very naughty age group, and the unknown behavior of the students has caused the teacher's feeling of stress. At this time, playing relaxing and soothing music in the teacher's office can relieve the teacher's tension; while the high school graduating class teacher faces the student group of a relatively mature age, the psychological pressure of the teacher stems from students' performance problems, and most of them are reflections on their own teaching methods. At this time, playing some exciting music will help eliminate graduating teachers' negative emotions, thereby enhancing their teaching morale.

### 4.3. The Effect of Music Therapy on Restaurant Employees

The chart shows that 15% of employees are satisfied with their work and 85% of employees feel average or dissatisfied. Restaurant employees are mainly faced with problems such as long working hours, high work intensity, and boring work tasks. Restaurant staff will have a sense of psychological pressure during long-term work. It would be very appropriate to apply music therapy programs to the psychological stress relief of restaurant employees. First of all, when employees are at work, the selected beautiful music is inadvertently heard in their ears, which allows employees to live in a comfortable and warm atmosphere and obtain a physically and mentally enjoyable experience. At the same time, music therapy also helps to improve the service level of restaurant staff. The main feature of music is rhythm. If its rhythm is unified with the human body's circadian rhythm, it will form a physiological resonance, and then people's body temperature, heartbeat, breathing, etc. may all change accordingly, which further allows people to have an enjoyable experience. The employees will also better demonstrate their service skills in the cheerful music. Second, music therapy can mobilize employees' work enthusiasm and improve their work attitude, which can further promote employees to provide consumers with satisfactory services. All in all, a good restaurant atmosphere is an important manifestation of the effect of restaurant management. Restaurant managers should effectively choose and apply the characteristics and functions of background music to create a good environment for the restaurant, so that consumers can also obtain physical and mental satisfaction.

## 5. Conclusion

Based on the satisfaction levels of the first three occupations, 15% of employees are satisfied with their jobs on average, while the remaining 85% feel generally or even dissatisfied with their jobs. The data prove that only a few employees have a sense of belonging and satisfaction with their work, so they all have different levels of work psychological pressure. The music therapy method can adopt targeted treatment programs for different occupations and ultimately reduce employees' psychological pressure. For example, music therapy can help medical staff relieve negative emotions and psychological pressure and keep them in a healthy mental state under high-intensity work content and work pressure. Music therapy can also help educators eliminate negative work pressure emotions, and even playing some exciting music will help strengthen the teaching morale of the teachers in the graduating class. Compared with traditional methods of solving employees' psychological stress, music therapy has the characteristics of being more efficient, more convenient, long-lasting, and low cost. Music therapy will also arouse the enthusiasm of the restaurant staff, improve their working attitude and their service level, and further promote the staff to provide satisfactory service to the consumers. As a crossdiscipline, music therapy can have a positive impact in many fields, especially in corporate applications, which can have a multifaceted positive impact on employees in the workplace. In the future, medical institutions or enterprises can make full use of music therapy to provide emotional regulation and psychological stress relief for employees or individuals. Increasing social competition in the future will also lead to more psychological pressure problems for employees in various industries. Music therapy theory and technology will be more perfect as researchers continue to join in. Music therapy can reduce the stress of employees in the workplace, promote their enthusiasm for work, and help employees to focus on work for a long time. This article uses case analysis and literature analysis methods and finally concludes that the use of music therapy will effectively improve the work efficiency of employees in the workplace.

## Figures and Tables

**Figure 1:** Impact of music therapy on employees' psychological and physical aspects.

**Figure 2:** Potential sources of work stress.

**Figure 3:** Satisfaction of employees in various occupations.

**Table 1:** Comparison table of general psychotherapy and music therapy.

	Effect	Treatment way	Scope of application	Cost
General psychotherapy	Less significant	Conversation, medication	Special population, small range	High
Music therapy	More significant	Have fun talking and music	Most people, wide group range	Low

## Data Availability

The datasets used and/or analyzed during the current study are available from the corresponding author on reasonable request.
